The article "Influence of Nutritional Support Program on Gastrointestinal Function, Complication Rate, and Prognosis in Elderly Sufferers with CI" was retracted in 2023. Reasons: unreliable results or conclusions; concerns about the data; concerns about the peer review; concerns about the citations.

# Influence of Nutritional Support Program on Gastrointestinal Function, Complication Rate, and Prognosis in Elderly Sufferers with CI

**DOI:** 10.1155/2022/3198272

**Published:** 2022-07-23

**Authors:** Huijuan Zhang, Jun Yang, Ying Xiong

**Affiliations:** ^1^Medical Experimental Center of Medical College, Jishou University, Xiangxi 416000, China; ^2^Department of Critical Care Medicine, Changde Fourth People's Hospital, Changde 415000, China; ^3^Department of Internal Medicine, Taoyuan Second People's Hospital, Changde 415000, China

## Abstract

To explore the effect of nutritional support program on gastrointestinal function, complication rate, and prognosis in elderly patients with cerebral infarction (CI), 200 elderly patients with CI from January 2020 to January 2021 are investigated in this study. The patients were randomly divided into a study set and a control group, with 100 cases in each set. All sets were given routine treatment, the control set was given parenteral nutrition support on a routine basis, and the study set was given enteral nutrition support on a routine basis. First, the clinical efficacy of the two sets after treatment was compared. Next, the constipation symptom score was adopted to compare the intestinal function of the two sets of patients before and after one month of treatment. The nutritional indicators, including serum albumin (ALB) and serum total protein (TP) levels, were compared between the two sets of patients before and after one month of treatment. Furthermore, the complications of the two sets of patients and the prognosis of the two groups of patients are analyzed. For elderly CI patients, enteral nutrition support therapy can significantly improve the clinical treatment effect, the gastrointestinal function, and nutritional index level. Also, it can reduce the incidence of complications and enhance the prognosis, survival rate, and quality of life.

## 1. Introduction

Cerebral infarction (CI) is caused by ischemia and hypoxia in sufferers due to blood circulation disorder, resulting in softening and necrosis of local brain tissue. With the aging of the population in my country, the prevalence of cerebrovascular diseases is increasing, and cerebral infarction accounts for about 70% to 80% of all cerebrovascular diseases [1]. Cerebrovascular disease has become a common disease in recent years, which has the characteristics of rapid onset, high mortality, high recurrence rate, and difficult therapy [2]. In medical research, it has always been a key research direction [3]. Cerebral infarction can cause physical sensory and motor dysfunction and even lead to the death of sufferers in a short period of time. Therefore, timely and accurate judgment of the location of cerebral infarction and the size of the lesion plays an important guiding role in clinical therapy [4]. However, some scholars believe that only 5% of sufferers with acute cerebral infarction receive thrombolytic therapy due to unclear early judgment and other reasons. Meanwhile, acute cerebral infarction is a very common clinical cerebrovascular disease, which can lead to the death of middle-aged and elderly people. Specifically, even if the therapy is timely and appropriate, most sufferers will leave sequelae of varying degrees, such as difficulty in movement, paralysis, language impairment, and intellectual impairment. The recurrence rate is extremely high, which is mentally and materially for the sufferers and their families bring a heavy burden [5]. With the development of medical technology, great progress has been made in the early diagnosis and therapy of cerebral infarction. However, sufferers often lose their ability to eat independently after therapy. Insufficient food intake leads to malnutrition and the decline of many bodily functions, resulting in poor health [6, 7]. Therefore, improving the prognosis of sufferers with cerebral infarction is still the focus of current clinical research. Nutritional support is to provide sufferers with necessary nutritional preparations through enteral and parenteral routes, but there are few comparative studies on the effects of enteral or parenteral nutrition [8]. The impact of serum nutritional indicators and prognosis in sufferers is reported as follows.

## 2. Related Work

After severe cerebral infarction, sufferers diagnosed with cerebral infarction often have impaired gastrointestinal function and difficulty in eating and swallowing and accompanied by mental retardation [9, 10]. It often leads to malnutrition, decreased immunity, and extensive increase in infectious diseases [11]. Among them, diseases such as hypoalbuminemia, high fever, and diarrhea are directly related to the mortality and complications of sufferers. Among the elderly with acute cerebral infarction, dietary and nutritional disorders are very common. The main reasons are as follows: (1) mental retardation or dysphagia following a traumatic event leading to eating problems; (2) the body is in a highly degenerative state at the time of cerebral infarction; (3) cerebral infarction with impaired gastrointestinal function, disease, and dyspepsia; and (4) older adults often share some commonalities that lead to imbalances [12]. Relevant studies have also confirmed that malnutrition is an independent risk factor for adverse outcomes in sufferers with cerebral infarction [13].

This study found that after 1 month of treatment, the nutritional indicators ALB and TP in the two sets were increased, and the research group was significantly higher than the control set (both *P* < 0.05). Important indicators can quickly show the nutritional changes of the patient's body. The Ruixian enteral nutrition emulsion used by this research team is mainly composed of maltodextrin, whey protein hydrolyzate, trace elements, dietary fiber,etc. Not only does it meet the nutritional needs of patients, but also helps maintain the intestinal function of patients [14]. Therefore, the nutrients in the serum of patients in the study set are higher than those in the control set. In addition, because CI patients have the characteristics of chronic high metabolic rate, poor nitrogen balance, and fast protein decomposition, timely enteral nutrition support can improve metabolism and stress levels, correct neurological function, effectively reduce protein synthesis, and maintain nutritional status. This study found that after 1 month of treatment, the constipation symptom scores of the two sets of patients decreased, and the constipation symptom scores of the study set were significantly lower than those of the control set, and the difference was statistically significant (all *P* < 0.05). The research set used an enteral nutrition pump to infuse nutrients to stimulate the intestinal mucosa, which can effectively improve gastrointestinal discomfort and the secretion of gastrointestinal hormones [15].

In medical practice, sufferers with cerebral infarction often have endocrine disorders, including hormone release and proteolysis in the hypothalamus. Because sufferers with this disease often have a certain degree of difficulty in eating, high energy consumption causes the body to regenerate and accelerate metabolism. Therefore, it is extremely important to provide sufferers with a balanced diet, but after the application of gastrointestinal nutritional support, some sufferers may experience mental disorders, vomiting, nausea, loss of appetite, poor nutrient absorption, etc., which will affect the sufferer's nutritional supplementation and later recovery. Therefore, it is extremely important to provide effective early enteral nutrition support for sufferers during hospitalization, and at the same time, it has a more positive therapeutic effect on sufferers with acute severe cerebral infarction [16, 17]. This study found that after therapy, a total of 6 sufferers in the study set had adverse reactions, which was notoriously lower than the 24 sufferers in the contrast set who had adverse reactions (*P* < 0.05). The survival rate of the study set was 93%, which was significantly higher than 76% of the contrast set; after 1 year of treatment, the quality of life scores of the two sets were increased, and the study set was significantly higher than the control set (*P* < 0.05). Due to enteral nutrition support, the food mix given to sufferers can be adjusted according to the important symptoms of the disease and the recovery of the body, and clinical courses are accepted to meet the requirements of clinical science. For sufferers with cerebral infarction and intestinal mucosal dysfunction, dietary intake is impaired, and the effect of regular water intake is negative, requiring professionals to adapt the diet in a balanced solution [18]. Enteral nutrition support not only supports and preserves the nutrients needed by the sufferer's body and supports therapy and the impact of disease but also reduces the risk of complications and maintains the normal function of the immune system [19, 20]. In addition, the food combination supported by enteral nutrition is rich in dietary fiber, which is easily ingested by the patients, improves the patient's diarrhea and constipation, can speed up the recovery of the disease, and ensure the patient's prognosis [21].

## 3. Proposed Methods

### 3.1. General Information

This study included 200 elderly sufferers with CI from January 2020 to January 2021, who were randomly divided into a study set and a contrast set, with 100 cases in each set. There were 46 males and 54 females in the research set, the age range was 51-68 years old, the average age was 61.35 ± 4.61 years old, the BMI was between 21 and 25 kg/m^2^, and the average was 23.47 ± 3.25 kg/m^2^. There were 47 males and 53 females, the age range was 50-69 years old, the average age was 61.59 ± 3.78 years old, the BMI was between 21 and 26 kg/m^2^, and the average was 24.17 ± 3.45 kg/m^2^; the two sets of sufferers were contrast. The general clinical data such as age and gender were *P* > 0.05, and there was no extensive disparity between the sets. All sufferers signed informed consent, and this study was approved by the Medical Ethics Committee of our hospital.

Inclusion criteria included are as follows: (1) consistent with the clinical diagnostic criteria and in line with the diagnostic criteria for cerebral infarction in the “China Guidelines for the Diagnosis and therapy of Acute Ischemic Stroke 2018,” (2) sufferers who can tolerate this study, (3) patients without gastrointestinal disease, (4) sufferers with high therapy enthusiasm and cooperated with physicians for therapy, and (5) sufferers and their families signed the informed consent.

Exclusion criteria included are as follows: (1) patients who do not meet the clinical diagnostic criteria and have not been diagnosed with acute cerebral infarction by physicians in our hospital, (2) pregnant and breastfeeding women, (3) patients with contraindications to enteral nutrition, (4) alcoholism and drug addicts, (5) combined with long-term malnutrition, (6) those with organic lesions in the liver and kidney, (7) those with gastrointestinal diseases, and (8) those who participated in other research trials other than this study.

### 3.2. Methods

Both sets were given conventional therapies such as intracranial pressure reduction, thrombolysis, antiplatelet aggregation, heparin, and neurotrophic agents. In special emergencies, hypertension therapy and blood sugar contrast could be given. Provide effective nursing care for all sufferers, monitor changes in sufferers' vital functions, maintain ward hygiene, contrast temperature and humidity, inform sufferers and their families of emergency situations such as prevention, and listen to psychological counseling; regularly communicate disease knowledge and successful case results with sufferers and their families, to enhance sufferer awareness of the disease and compliance with therapy. During taking the medicine, it is necessary to follow the medication instructions, strictly follow the doctor's instructions, contrast the time and dosage of the medication, record the changes in the sufferer's body during therapy, and inform the sufferer and family about the side effects of the drug. For rehabilitation training for sufferers with special needs, the affected limbs should be replaced regularly to assist passive learning, such as height, extension and rotation, and internal and external conversion. Prevent disease, help sufferers to change frequently, maintain personal hygiene, remind family members to complete turning over for sufferers regularly, and use air mattresses, turning pads, and other appliances to prevent pressure ulcers and infection.

For contrast set, provide parenteral nutrition support in addition to routine care. Parenteral nutrition support included energy consumption measured on an H-B scale, intravenous infusion of artificial nutrients such as glucose, amino acids, and fat milk, with an adult calorie target of 25-30 kcal/kg, and administration of 50.0% basal body weight 2 days before treatment and subsequent increase to full volume.

For research set, enteral nutrition support was supplemented on the basis of conventional therapy. Enteral nutrition support includes the following: measuring energy consumption according to H-B scale, using enteral nutrition pump for infusion, and the nutritional agent is enteral nutrition emulsion (trade name: Ruixian; manufacturer: Fresenius Kabi Huarui Pharmaceutical Co., Ltd.; National Medicine Zhunzi H20040188). Patients were administered by tube feeding, and the daily dose was calculated by weight and nutritional status. Based on weight, nutritional status, and energy requirements, it is 20 ml (30 kcal) to 30 ml (45 kcal)/kg per day. When administered in tube feeding, the dose should be increased gradually, at a rate of about 20 ml an hour on the first day. After that, increase 20 ml one hour day by day until the daily dose required by the patient is reached. The maximum drip rate is 125 ml for one hour, and the infusion rate is adjusted by pump.

### 3.3. Observation Indicators

#### 3.3.1. Clinical Efficacy

According to the sufferer's neurological deficit and the degree of disability, the efficacy of the sufferer is judged, among which recovery is as follows: the neurological deficit score is reduced to more than 91%, and the degree of disability is 0; markedly effective: the neurological deficit score is 46-90%, and the degree of disability is 1-3; progress: the neurological deficit score is 18-45%; ineffective: the neurological deficit score is below 17%. Total effective can be defined as rate = (cure + marked effect + progress)/total number of cases × 100%.

#### 3.3.2. Intestinal Function

Before therapy and after 1 month of therapy, constipation symptom scores include constipation symptom score and evaluation method of constipation efficacy. The constipation symptoms and efficacy evaluation questionnaire developed by the Anorectal Surgery Scientific set of the Chinese Medical Association Surgery Branch were used, including defecation difficulty, stool character, defecation time, feeling of falling and incompleteness, defecation in the six aspects of frequency, and abdominal distension. Each item is scored from 0 to 3 points.

#### 3.3.3. Nutritional Indicators

The serum nutritional indicators before therapy and 1 month after therapy are chosen. Fasting venous blood was centrifuged to take the supernatant using an automatic biochemical analyzer (manufacturer: Shenzhen Mindray Medical Electronics; model: BS-2000M) to detect the levels of serum albumin (albumin, ALB) and serum total protein (TP) in sufferers.

#### 3.3.4. Complications

Complications in the two sets were contrast. They include pulmonary infection, electrolyte imbalance, and gastrointestinal bleeding. The total incidence of complications (%) is defined as the number of complications/total number × 100%.

#### 3.3.5. Prognosis

Contrast the prognosis of the two sets of sufferers. The two sets were followed up for one year, and the survival rates (survival curves) of the two sets were recorded; MOS item short from health survey, SF-36. The scale is a 36-item structured questionnaire that includes physiological function (PF), role-physical (RP), body pain (BP), general health (GH), vitality (VT), social functioning (SF), role-emotional functioning (RE), and mental health (MH). 36 items in eight dimensions comprehensively summarize the life quality of the subjects. Total score (TS) adopts the unified standard score in China, ranks each item, and then accumulates the item scores of each dimension. For the scale, the original score is calculated first, and then, the converted score is calculated using the standardized formula. The formula is as follows: conversion score = (actual score − the lowest possible score in this aspect)/the difference between the highest possible score and the lowest possible score in this aspect ×100. Conversion score for each dimension and each field is 100, and the lowest score is 0. The higher the score, the better the quality of life.

### 3.4. Statistical Methods

In this study, all the data were organized, and a corresponding database was established for it, and all the databases were entered into SPSS 26.0 for data processing, and the measurement data was tested for normality, expressed as *x* ± *s*, consistent with positive. The independent samples *t* test was used for the data between sets, the paired samples *t* test was used for the data within the set, and the Mann-Whitney *U* test was used for nonnormality; the rate was expressed as %, and the test was *χ*^2^. The test was used to analyze the prognosis and survival rate. When *P* < 0.05, the disparity between the data was considered to be statistically extensive.

## 4. Results

### 4.1. Contrast of Clinical Efficacy between the Two Sets of Sufferers

The clinical effective rate of sufferers in the study set was 95.00%, which was notoriously higher than 73.00% in the contrast set, and the disparity was statistically extensive (*P* < 0.05), as shown in Table 1.

### 4.2. Contrast of Intestinal Function Changes between the Two Sets at Different Time Points

Before treatment, there was no significant difference in constipation symptom scores between the two groups (*P* > 0.05). After 1 month of treatment, the constipation symptom scores of the two groups were decreased, and the constipation symptom scores of the study group were significantly lower than those of the control group, and the difference was statistically significant (*P* < 0.05), as shown in Table 2. The symbol ∗ indicates that contrast with before therapy, *P* < 0.05, the disparity is statistically extensive.

### 4.3. Contrast of Changes in Nutritional Indicators between the Two Sets at Different Time Points

Before therapy, there was no extensive disparity in nutritional indexes ALB and TP between the two sets (*P* > 0.05). After 1 month of treatment, the nutritional indexes ALB and TP in the two sets were increased, and the study set was significantly higher than the control set (all *P* < 0.05), as shown in Table 3. The symbol ∗ indicates that contrast with before therapy, *P* < 0.05, the disparity is statistically extensive.

### 4.4. Contrast of Complications between the Two Sets

After therapy, a total of 6 sufferers in the study set had adverse reactions, which was notoriously lower than the 24 sufferers in the contrast set who had adverse reactions (*P* < 0.05), as shown in Table 4 and Figure 1.

### 4.5. Contrast of the Survival of the Two Sets

Two sets of sufferers were followed up for one year, the follow-up time ended in January 2022. The survival rate of the study set was 93% (93/100), which was notoriously higher than that of the contrast set, 76% (76/100). Also, the disparity was statistically extensive (*P* < 0.05), as shown in Figure 2.

### 4.6. Contrast of the Quality of Life between the Two Sets at Different Time Points

Before intervention, the scores of quality of life of the two sets were lower, and the disparity was not statistically extensive (*P* > 0.05). After 1 year of therapy, the scores of quality of life of the two sets were increased, and the study set was notoriously higher than contrast set (*P* < 0.05), as shown in Table 5. The symbol ∗ means contrast with before therapy, & means contrast with contrast set, *P* < 0.05, and the disparity was statistically extensive.

## 5. Conclusions

In this study, 200 elderly patients with CI from January 2020 to January 2021 are investigated to explore the effect of nutritional support program on gastrointestinal function, complication rate, and prognosis in elderly patients with cerebral infarction (CI). For elderly CI sufferers, enteral nutrition support therapy can notoriously enhance the clinical therapy effect, improve the level of gastrointestinalfunction and nutritional index of patients, reduce the occurrence of complications, improve the prognosis of patients with quality of life, which is worthy of clinical application.

## Figures and Tables

**Figure 1:** Contrast of the incidence of adverse reactions between the two sets.

**Figure 2:** Contrast of survival in the two sets within one year.

**Table 1:** Contrast of clinical efficacy between the two sets of sufferers.

Set	Get well	Efficient	Progress	Invalid	Total efficiency
Contrast set (*n* = 100)	23 (23.00)	26 (26.00)	24 (24.00)	27 (27.00)	73 (73.00)
Study set (*n* = 100)	59 (59.00)	21 (21.00)	15 (15.00)	5 (5.00)	95 (95.00)
*χ* ^2^					16.893
*P*					<0.001

**Table 2:** Contrast of intestinal function changes between the two sets at different time points.

Set	Constipation symptom score (points)	
	Before therapy	1 month after therapy
Contrast set (*n* = 100)	11.01 ± 2.96	8.21 ± 1.63^∗^
Study set (*n* = 100)	10.85 ± 2.89	5.19 ± 1.06^∗^
*t*	0.951	14.563
*P*	0.218	<0.001

**Table 3:** Contrast of changes in nutritional indicators between the two sets at different time points.

Set	ALB (g/l)		TP (g/L)	
	Before therapy	1 month after therapy	Before therapy	1 month after therapy
Contrast set (*n* = 100)	26.49 ± 1.53	31.41 ± 4.51^∗^	60.96 ± 4.29	64.12 ± 4.33^∗^
Study set (*n* = 100)	26.75 ± 1.45	36.15 ± 5.27^∗^	61.53 ± 4.17	70.17 ± 4.53^∗^
*t*	0.631	11.851	0.775	10.571
*P*	0.501	<0.001	0.453	<0.001

**Table 4:** Contrast of complications between the two sets.

Set	Lung infection	Electrolyte imbalance	Gastrointestinal bleeding	Total incidence
Contrast set (*n* = 100)	8 (8.00)	7 (7.00)	9 (9.00)	24 (24.00)
Study set (*n* = 100)	2 (2.00)	2 (2.00)	2 (2.00)	6 (6.00)
*χ* ^2^				15.417
*P*				<0.001

**Table 5:** Contrast of the quality of life between the two sets at different time points.

Project	Set	Before therapy	1 year after therapy
PF	Study set (*n* = 100)	52.56 ± 4.25	85.56 ± 5.26^∗^^&^
	Contrast set (*n* = 100)	53.66 ± 4.19	65.33 ± 5.17^∗^
RP	Study set (*n* = 100)	62.23 ± 4.79	89.42 ± 3.38^∗^^&^
	Contrast set (*n* = 100)	62.81 ± 4.91	70.10 ± 3.35^∗^
BP	Study set (*n* = 100)	76.56 ± 3.15	83.34 ± 4.57^∗^
	Contrast set (*n* = 100)	76.35 ± 3.56	80.55 ± 4.79^∗^
GH	Study set (*n* = 100)	75.31 ± 5.12	86.69 ± 3.03^∗^^&^
	Contrast set (*n* = 100)	75.81 ± 5.62	82.10 ± 3.34^∗^
VT	Study set (*n* = 100)	55.75 ± 5.31	63.17 ± 3.36^∗^
	Contrast set (*n* = 100)	56.24 ± 5.34	60.67 ± 3.17^∗^
SF	Study set (*n* = 100)	55.99 ± 3.16	66.15 ± 3.04^∗^^&^
	Contrast set (*n* = 100)	55.60 ± 3.32	61.65 ± 3.13^∗^
RE	Study set (*n* = 100)	74.74 ± 5.18	82.75 ± 3.51^∗^
	Contrast set (*n* = 100)	75.10 ± 5.57	80.22 ± 2.06^∗^
MH	Study set (*n* = 100)	68.12 ± 5.68	73.19 ± 3.49^∗^
	Contrast set (*n* = 100)	67.17 ± 5.70	71.75 ± 3.66^∗^

## Data Availability

The simulation experiment data used to support the findings of this study are available from the corresponding author upon request.

## References

[1] Zhu X. L., Sun F. H. (2019). Application effect of early enteral nutrition nursing intervention on sufferers after massive cerebral infarction decompression. *Clinical Research and Practice*.

[2] Yuan T., Zeng G., Yang Q. (2021). The effects of total enteral nutrition via nasal feeding and percutaneous radiologic gastrostomy in patients with dysphagia following a cerebral infarction. *American Journal of Translational Research*.

[3] Xian H. (2019). Effect of early enteral nutrition nursing intervention on the prognosis of sufferers after extensive cerebral infarction decompression. *Chinese Journal of Practical Nervous Diseases*.

[4] Merkler A. E., Alakbarli J., Barbar T. (2020). Associations between the size and location of myocardial infarction and cerebral infarction. *Journal of the Neurological Sciences*.

[5] Wang L. F., Tang X. H., Zhang X. X. (2019). Influencing factors of misinhalation in sufferers with severe cerebral infarction undergoing enteral nutrition support and nursing strategies. *Hainan Medical Journal*.

[6] Xia Y., Sheng-Nan W. U., Diao Y. F., Li Y. L. (2019). Effect of low calorie and high protein enteral nutrition on nutritional indexes and complications in sufferers with acute cerebral infarction. *Parenteral& Enteral Nutrition*.

[7] Cheng S., Neurology D. O. (2019). Application of doctor-nurse integration in nursing care of enteral nutrition supporting for critically ill sufferers in neurology intensive care unit. *Nursing of Integrated Traditional Chinese and Western Medicine*.

[8] Bin P., Bo W. (2019). Guidelines for the diagnosis and treatment of acute Ischemic stroke in China 2018. *Chinese Journal of Neurology*.

[9] Cheng Y., Dai Y., Neurology D. O. (2018). Evaluation of early enteral nutrition support in sufferers with acute cerebral infarction. *Chinese Journal of Practical Nervous Diseases*.

[10] Lian X., Wu M., Fan H., Zhang Y., Sun P. (2020). Wernicke's encephalopathy due to malnutrition and parenteral nutrition in a sufferer with cerebral infarction: a case report. *Medicine*.

[11] Zhang H. R., Li W. H., Li X. (2019). Clinical observation of early comprehensive rehabilitation therapy on acute cerebral infarction. *China & Foreign Medical therapy*.

[12] Jukic N., Gagliardi C., Fagnani D., Venturini C., Orlandoni P. (2017). Home Enteral Nutrition therapy: Difficulties, satisfactions and support needs of caregivers assisting older patients. *Clinical Nutrition*.

[13] Wang J. X., Wang Y. Y., Meng L. L. (2022). The application effect of early different enteral nutrition support in sufferers with severe cerebral infarction. *Journal of Integrated Traditional Chinese and Western Medicine Cardiovascular and Cerebrovascular Diseases*.

[14] Yang H. Y., Yuan F., Xie H. W. (2021). Application of ‘Internet+’ continuous nutrition management model in home enteral nutrition for sufferers with cerebral infarction and dysphagia. *PLA Nursing Journal*.

[15] Li X. L., Han L. (2020). Effects of glutamine combined with sequential enteral nutrition therapy on nutritional status and prognosis of sufferers with severe cerebral infarction. *Anhui Medicine*.

[16] Zhu Y. T., Liu Z. Y., Wang F. Y. (2020). The clinical value of precision nursing in enteral nutrition support for sufferers with cerebral infarction. *Western Medicine*.

[17] Liu L. J. (2020). Effect of early enteral nutrition support on clinical outcomes of sufferers with acute severe cerebral infarction. *Journal of Chengdu Medical College*.

[18] Zhou L., Hua J., Shen L. Y. (2020). Discussion on the efficacy and mechanism of intensive probiotic regimen assisted enteral nutrition in the therapy of severe acute cerebral infarction. *Journal of Integrated Traditional Chinese and Western Medicine Cardiovascular and Cerebrovascular Diseases*.

[19] Jo H. J., Shin D. B., Koo B. K., Ko E. S., Yeo H. J., Cho W. H. (2017). The impact of multidisciplinary nutritional team involvement on nutritional care and outcomes in a medical intensive care unit. *European Journal of Clinical Nutrition*.

[20] Jiao M. Z., Ma H. G., Lu B. (2020). Effects of early enteral nutrition on the structure and nutritional status of intestinal flora in sufferers with acute cerebral infarction. *China Journal of Microecology*.

[21] Yan J., Yao Y., Yan S., Gao R., Lu W., He W. (2020). Chiral protein supraparticles for tumor suppression and synergistic immunotherapy: an enabling strategy for bioactive supramolecular chirality construction. *Nano Letters*.

